# Slug contributes to cancer progression by direct regulation of ERα signaling pathway

This article has been retracted.

**DOI:** 10.3892/ijo.2015.2878

**Published:** 2015-02-05

**Authors:** YOUQIANG LI, YANYUAN WU, THOMAS C. ABBATIELLO, WARREN L. WU, JU RI KIM, MARIANNA SARKISSYAN, SUREN SARKISSYAN, SEYUNG S. CHUNG, YAHYA ELSHIMALI, JAYDUTT V. VADGAMA

**Affiliations:** 1 Division of Cancer Research and Training, Charles R. Drew University of Medicine and Science, Los Angeles, CA 90059, USA; 2 University of California at Los Angeles David Geffen School of Medicine, and UCLA Jonsson Comprehensive Cancer Center, Los Angeles, CA 90024, USA

**Keywords:** Slug, breast cancer, prostate cancer, ERα, DNA binding

## Abstract

Hormone therapy targeting estrogen receptor α (ERα) is the most effective treatment for breast cancer. However, this treatment eventually fails as the tumor develops resistance. Although reduced expression of ER-α is a known contributing factor to endocrine resistance, the mechanism of ER-α downregulation in endocrine resistance is still not fully understood. The present study shows that Slug has an inverse relationship with ERα in breast and prostate cancer patient samples. Also the inhibition of Slug blocks mammary stem cell activity in primary mammary epithelial cells. We hypothesize that Slug may be a key transcription factor in the regulation of ERα expression. To understand the Slug-ERα signaling pathway, we employed resistant cell line MCF-TAMR (ERα relatively negative) derived from its parental MCF-7 (ERα positive) cell line and assessed changes in cell phenotype, activity and response to therapy. Conversely, we performed knockdown of Slug in the high-Slug expressing cell line MDA-MB-231 and assessed reversal of the mesenchymal phenotype. Microarray analysis showed that Slug is overexpressed in high grade breast and prostate cancer tissues. Additionally, Slug overexpression leads to drug resistance. Furthermore, we demonstrated that Slug binds directly to ERα promoter E-boxes and represses ERα expression. This resulted in decrease in epithelial-to-mesenchymal transition in cancer cells. These findings demonstrate that Slug, by regulation of ERα expression, contributes to tumor progression and could serve as an important target for cancer therapy.

## Introduction

Mechanisms of drug resistance include many factors, including decreased intracellular drug concentration which could result from increased drug efflux via the ATP binding cassette (ABC) transporters such as MDR-1/P-glycoprotein. In addition, decreased conversion of the drug to an active form, and altered amount of drug target or altered target type (1,2) could influence resistance. ER-α is a hormone-dependent nuclear transcription factor that is expressed in ~70% of breast tumors. Tamoxifen treatment decreases cancer recurrence by 50% and reduces the annual breast cancer death rate by 25–30% (3). However, many patients with ERα positive breast cancer eventually acquire resistance to tamoxifen (3).

Epithelial-mesenchymal transition (EMT) is a biological process where cells lose their epithelial characteristics and acquire a mesenchymal phenotype with increased migratory behavior. EMT could lead to increase in motility, invasivenes-sand metastatic capabilities of cancer cells (4,5). Recently, mesenchymal-like characteristics have been associated with resistance to erlotinib, gefitinib, and cetuximab treatment in non-small cell lung cancer, head and neck squamous cell carcinoma, pancreatic cancer and hepatocellular carcinoma (6–9).

Tumors arise in tissues and organs that undergo constant remodeling and regeneration. We hypothesized that tumor initiation and progression are steps driven by cancer stem cells (CSCs). Cancer stem cells have been isolated and characterized initially from leukemia and subsequently from solid tumors, including brain, breast, prostate, colon and liver cancer (10–14). In the cancer-stem-cell model of drug resistance, tumors may express a population of drug-resistant pluripotent cells that can survive chemotherapy and subsequently regrow into metastatic tumors (15,16).

Slug (Snail2), a C2H2-type zinc finger transcription factor, also an EMT marker, has been identified in aggressive cancers and is correlated with worse clinical outcomes in colon and ovarian cancers (17,18). Slug and Sox9 cooperatively determine the mammary stem cell state (6) and Slug is highly expressed in triple-negative breast cancer (19). However, the role of Slug in the development breast cancer drug resistance is unclear.

The mechanistic relationship between EMT, loss of cell polarity, and CSC characteristics remains an open question in cancer biology. In the present study, we found that Slug is overexpressed in high grade breast and prostate cancers. We also uncovered *de novo* function of Slug, where it directly binds to E-boxes of ERα promoter region and decreases ERα synthesis. In addition, Slug contributes to drug resistance and EMT phenotype in breast cancer cell lines. Slug may play an important role as a predictive marker for cancer progression and could be targeted for therapy against tumor resistance and metastasis.

## Materials and methods

### Cell lines, DNA constructs and antibodies

Human breast cell lines, MCF10A (cat. CRL-10317), MCF12A (cat. CRL-10782), MCF7 (cat. HTB-22), MDA-MB-231 (cat. HTB-26), and prostate cancer cell line LNCap (cat. CRL-1740) were purchased from the American Type Culture Collection (ATCC, Manassas, VA, USA) and cultured in DMEM/F-12 50/50 media (cat. 11320-033; Thermo Fisher Scientific, Waltham, MA, USA) supplemented with 10% fetal bovine serum (cat. 10437-028; Life Technologies, Grand Island, NY, USA) 1% penicillin/streptomycin (cat. 15070-063; Life Technologies). MCF10A and MCF12A cells were cultured in DMEM/F-12 50/50 media supplemented with 5% horse serum (cat. 26050070; Life Technologies), 20 ng/ml EGF (cat. PHG0311L; Life Technologies) and 10 μg/ml insulin (cat. I0516; Sigma-Aldrich, St. Louis, MO, USA). The MCF7-TAMR (MCF7 tamoxifen resistance cell line, a gift from Dr Kent Osborne, Baylor College of Medicine, Houston, TX, USA) was generated from MCF7 cells grown in phenol red-free DMEM/F-12 media (cat. 21041-025; Life Technologies) supplemented with 10% charcoal/dextran-stripped (CDS) FBS (cat. 12676-029; Life Technologies) and incrementally treated and cultured in increasing concentrations of tamoxifen (cat. T5648; Sigma-Aldrich). LNAI (LNCaP androgen independent) cell line was generated from LNCaP cells grown in phenol red-free DMEM/F-12 50/50 supplemented with 10% CDS FBS and antibiotics for a long period of time. Human snail homolog 2 (*Drosophila*) (SNAI2/SLUG, NM_003068) cDNA ORF clone (cat. RG202363) and pCMV6-AC-GFP vector (cat. PS100010) were purchased from OriGene (Rockville, MD, USA). MCF7 cells were stably transfected with either the SNAI2 human cDNA ORF clone (MCF7/Slug) or pCMV6-AC-GFP vector (MCF7/V) using Lipofectamine 2000 (cat. 11668-019; Life Technologies). The SLUG ShRNA, purified plasmid DNA target-SLUG silencing and Control shRNAs (sc-38393-SH) were purchased from Santa Cruz Biotechnology (Santa Cruz, CA, USA). Transfection of MDA-MB-231 cells was performed using the SLUG shRNA (MDA/shSlug) and control shRNAs (MDA/shCon) using the shRNA plasmid transfection reagent (sc-108061; Santa Cruz Biotechnology) and following the manufacturer’s protocol and selected under puromycin (10 μg/ml) (cat. A1113802; Life Technologies) treatment.

### Estrogen induction assay

β-estradiol (E2) was purchased from Sigma (E8875; Sigma-Aldrich). The cells were cultured in DMEM/F-12 50/50 with 10% CDS FBS, incubated with 5% CO_2_/air at 37°C for 2 days, and then 10 nM E2 was supplemented in the media containing 10% CDS FBS for 24, 48 and 72 h. Cell growth was measured using MTT assay as previously described (20).

### Immunoblotting assay

Total protein lysates were prepared using RIPA buffer (cat. 89900; Thermo Fisher Scientific). Nuclear proteins were isolated using NE-PER nuclear and cytoplasmic extraction reagents (cat. 78833; Thermo Fisher Scientific) and 30 μg of protein were separated on 4–15% SDS-PAGE (#456-1086; Bio-Rad Laboratories, Hercules, CA, USA) and transferred onto PVDF membrane (#162-0177; Bio-Rad Laboratories). Membranes were probed using the following antibodies: β-actin (sc-69879; 1:2,000 dilution), androgen receptor (sc-7305; 1:1,000), c-Myc (sc-42; 1:1,000), CD24 (sc-7034; 1:500), CD44 (sc-59909; 1:500), ER-α (sc-8005; 1:1,000), EGFR (sc-03; 1:500), Laminin A/C (sc-6215; 1:1,000), Oct-3/4 (sc-8629; 1:500), Slug (sc-15391; 1:500), Sox2 (sc-20088; 1:500), Twist (sc-15393; 1:1,000) and Vimentin (sc-5565; 1:1,000) from Santa Cruz Biotechnology. The image was developed with the Super Signal West Pico Chemiluminescent (cat. 34077; Thermo Fisher Scientific), and visualized by Bio-Rad ChemiDoc XRS imagining system.

### Transwell cell migration assay

Transwell assay was performed using Boyden chambers (cat. CBA110; Cell Biolabs, Inc., San Diego, CA, USA) containing polycarbonate membranes. Briefly, cells were serum starved overnight and then 100 μl of 50,000 cells in serum-free media were added to the upper chamber and 300 μl of the appropriate media with 10% FBS was added to the lower chamber. The Transwell was incubated for 48 h at 37°C. Non-migratory cells on the upper membrane surface were removed with a cotton swab, and the migratory cells on the undersurface of the membrane were fixed and stained with 0.2% crystal violet (cat. c581-25; Thermo Fisher Scientific) for 20 min at room temperature. The numbers of invaded cells were counted under light microscope (Leica Microsystems, Inc., Buffalo Grove, IL, USA). The average number of invaded cells was calculated from three random regions, and images were captured by Olympus digital camera (Olympus BioScapes, Allentown, PA, USA) under the light microscope.

### Three dimensional Matrigel assay

Matrigel (cat. A1413201; Life Technologies) was spread as a thick layer on a 24-well plate (cat. 08-772-1; Thermo Fisher Scientific) and allowed to polymerize at 37°C for 15 min. Cells (2×10^4^/well) were plated on top of the pre-coated Matrigel wells and incubated at 37°C until fully settle, and then growth media containing 5% Matrigel was added. The growth media with Matrigel was changed every 2 days. Cells were grown for 15 days and the images of representative fields were taken by Olympus digital camera (Olympus BioScapes) under the light microscope.

### Immunofluorescence

Cells were fixed using 4% formaldehyde (SF96-20; Thermo Fisher Scientific) for 10 min at room temperature and then blocked with 2.5% normal house serum blocking solution (cat. S-2012; Vector Laboratories, Inc., Burlingame, CA, USA). The cells were then incubated with ER-α (PA0151; Leica Microsystems) and Slug (sc-15391, 1:500; Santa Cruz Biotechnology) primary antibodies for 1 h at room temperature followed by incubation with FITC conjugated second antibodies (anti-mouse IgG-FITC: sc-2010, or anti-rabbit IgG-FITC: sc-2012 from Santa Cruz Biotechnology) for 30 min. Cell nuclei were counterstained using 4′,6-diamidino-2-phenylindole (DAPI) (cat. D9542; Sigma-Aldrich). Imaging was taken by a digital camera microscope (Olympus BioScapes) under the light microscope.

### Real-time PCR (q-PCR)

RNA was isolated from cultured cells using RNeasy Mini kit (cat. 74104; Qiagen, Valencia, CA, USA). Synthesis of cDNA was performed using 1 μg of RNA with ThermoScript RT-PCR system (cat. 11146-016; Life Technologies). The q-PCR was performed using GeneRead qPCR SYBR-Green/Fluor Master Mix (cat. 180830; Qiagen) with the Real-Time PCR Detection system (iCycler; Bio-Rad Laboratories). Primer sequences used for RT-PCR can be found in Table I.

### Chromatin immunoprecipitation (ChIP) assay

ChIP assay was performed using EMD Millipore ChIP Assay kit (cat. 17-295) according to the manufacturer’s suggested protocol (Millipore, Billerica, MA, USA). Cells were cross-linked using 1% formaldehyde solution (cat. 252549; Sigma-Aldrich). Immunoprecipitation was performed using 1 μg of anti-Slug antibody, or normal goat IgG (cat. sc-2028; Santa Cruz Biotechnology). Quantitative real-time PCR was performed on isolated DNA using GeneRead qPCR SYBR Green/Fluor Master Mix (cat. 180830; Qiagen) with the E-box primers. The primers sequences contain the specific binding site on ERα promoter and are listed in Table I.

### Tumorigenicity in nude mice

The experimental animals used in the present study were approved by the Institutional Animal Care and Use Committee (IACUC) at Charles R. Drew University of Medicine and Science at USA. The animal research was performed according to the internationally recognized guidelines on animal welfare.

Ten 7-week-old female nude mice (Harlan Laboratories, Livermore, CA, USA) were divided into two groups with 5 in each group. Total 1×10^6^ cells in 0.1 ml of PBS containing 50% Matrigel were injected into the top mammary fat pad of the 7-week-old female nude mice. Tumor size was measured weekly in 2 dimensions with calipers. Tumor volume (V) was determined according to the formula ½ (length × width^2^). Two sample t-tests were used to compare tumor volumes between the groups.

### Immunohistochemistry of tissue microarray (TMA)

The TMA was constructed from specimens obtained from an ongoing breast cancer study conducted by the Division of Cancer Research and Training at Charles R. Drew University of Medicine and Science (CDU) in Los Angeles, CA, USA. The study on human samples was approved by the Institutional Review Board of CDU. Written informed consent was obtained from each subject.

The breast TMA was constructed similarly to the array previously described (21). Briefly, histology of each specimen from haematoxylin and eosin (H&E) stained sections were carefully reviewed and marked on corresponding individual paraffin blocks by a clinical pathologist. Three 1.0-mm tissue cores were taken from each selected specimen and placed in one receiver arrayed paraffin block (cat. IW-125; IHC World LLC, Woodstock, MD, USA). Non-neoplastic breast tissue cores were also included in each tissue microarray block.

Prostate cancer TMA slide (PR951) used in the present study was purchased from US Biomax Inc (Rockville, MD, USA), a commercial vendor of biospecimens. The prostate cancer TMA is comprised of 95 cores from 48 cases including malignant tissues and normal tissues. The information of Gleason score at surgery for the malignant tumor tissues was obtained from Biomax at the time of purchasing.

### Statistical analysis

Statistical analysis was performed with the SPSS statistical package (version 11.0 for windows; IBM). The Student’s t-test was used to examine the variance between different treatment groups. P-values <0.05 were considered statistically significant.

## Results

### ERα is downregulated in tamoxifen resistant MCF7 cells

Breast cancer is the most common malignant cancer type in women (22). Breast cancer requires gonadal steroids for its development and it is typically hormone-dependent. Receptor antagonists of the ERα subtype, such as tamoxifen, are commonly used to block ERα action in breast cancer (23). The receptor antagonist treatment is an effective initial approach for ERα-positive breast cancer patients, however, resistance eventually occurs. The development of tamoxifen resistance in MCF-TAMR cell line has been demonstrated *in vitro* (Fig. 1a). MCF-TAMR shows decreased sensitivity to tamoxifen (Fig. 1b) and the cell growth was independent of added 17β-estradiol (E2) (Fig. 1c). The expression level of ERα was reduced in MCF-TAMR cells compared to MCF7 cells (Fig. 1d–f). Downregulation of ERα may be a reason for tamoxifen resistance. MCF-TAMR has acquired invasive characteristics as demonstrated by the invasion assay (Fig. 1g and h).

### Slug has inverse relationship with ERα and is correlated with cancer progression in breast and prostate cancer

Developmental studies have demonstrated that master transcription factors, such as Oct4 and c-Myc (24) play a central role in determining cellular states. These transcription factors may also be very important for tumor development and drug resistance. We examined the mRNA expression of several transcription factors, including those that are associated with stem-like properties. Our data show a significant upregulation of Slug, Twist, c-Myc, c-Jun, Sox2 and Oct4 in MCF-TAMR cells (Fig. 2a). Noatbly, wild-type MCF7 cells treated with tamoxifen showed ~2-fold increase in Slug, c-Myc and c-Jun. ERα, AR and β-catenin were slightly downregulated in both MCF7 cell types treated with tamoxifen as well as in MCF-TAMR cells. Only Sox9 was significantly downregulated in MCF7 cells treated with tamoxifen (Fig. 2a). The importance of Slug, c-Myc and c-Jun increase in response to tamoxifen treatment in MCF7 cells needs further examination. The continued upregulation of these three transcription factors in MCF-TAMR suggests they may play a role in the drug resistance.

Recent studies suggest that Slug functions as a transcriptional repressor and plays an important role in embryonic and breast tissue development (6,25) as well as in cancer (26,27). The present study shows that Slug has an inverse relationship to ERα in MCF7 and MDA-MB-231 breast cancer cell lines (Fig. 2b and c). We examined this relationship in patient samples. Fig. 2d and g shows the expression of Slug and ERα analyzed by immunohistochemistry (IHC) in breast tissues from breast cancer patients with known clinical diagnosis and follow-up. Each sample/spot on the tissue microarray (TMA) platform represented different cancer subtype and stage. Our data show low Slug expression in normal and ductal carcinoma *in situ* (DCIS) breast cancer samples, while Slug expression was significantly increased in infiltrating ductal carcinoma (IDC) (Fig. 2d and e). An inverse correlation is shown between Slug and ERα expression in Fig. 2f and g.

To understand the function of Slug expression in another type of cancer, we examined Slug expression in prostate cancer, which is also commonly treated with anti-hormonal agents and/or androgen deprivation (28) and similarly develops resistance to therapy. Notably, ERα expression decreased significantly in prostate cancer tissues compared to normal prostate tissue. There was an inverse relationship between loss of ERα and increase in Slug expression in prostate cancer tissues with increasing Gleason score (8 to 10) and in metastatic cancer tissues, compared to low Gleason score (6 to 7) and normal samples (Fig. 3a and b). This inverse correlation between Slug and ERα expression was similar to the breast cancer tissue microarray (TMA) (Figs. 2f and 3a and b). As per the TMA data, there were three prostate cancer-related deaths and Slug expression was significantly high in these patients (Fig. 3c). Notably, in both breast and prostate cancers Slug was overexpressed during disease progression. Other groups have also reported that Slug expression is correlated with worse clinical outcome in hepatocellular carcinoma and colorectal cancer (26,27). Thus, Slug may be a predictive biomarker for metastatic cancers with poor outcome. Next, we sought to determine the mechanisms by which Slug could contribute to cancer progression.

### Slug binds to E-boxes in the promoter region of ERα gene

It is well established that cancer can be considered a disease of cell de-differentiation (29–31). ERα is a marker for terminal differentiated non-cancer normal breast luminal cells (32). Negative correlation between expression of Slug and ERα made us conclude that Slug may play a central role in cell differentiation. To determine whether Slug regulates ERα expression, Slug and ShSlug plasmid transfection analysis was performed in MCF7 cell line (Slug-negative/ERα-positive) and MDA-MB-231 cell line (Slug-positive/ERα-negative) lines (Fig. 2c). Transiently overexpressed Slug successfully reduced ERα levels in MCF7 cells whereas downregulation of Slug increased the ERα expression in MDA-MB-231 cells (Fig. 4a and b). Thus, when Slug is highly expressed in ERα-negative breast cells, ERα synthesis is reduced. The Slug and ERα expression were observed in two normal breast cell lines: MCF10A and MCF12A. MCF10A (high expression of Slug and low expression of ERα) showed no signs of terminal differentiation or senescence (33). MCF12A (low expression of Slug and higher expression of ERα) is a differentiated breast luminal cell (34,35) (Fig. 4c). Knockdown of Slug (ShSlug) in MCF10A cells increased ERα expression while overexpressed Slug in MCF12A cells decreased ERα expression (Fig. 4d and e). These combined results show that Slug can regulate ERα expression in both normal and cancer breast cells.

ERα genomic amplification is observed in breast cancer patients overexpressing ERα (36). We determined that genomic ERα is amplified in MCF7, MCF-TAMR and MDA-MB-231 cell lines compared to normal epithelial breast cell lines (Fig. 4f). In addition, there was no significant difference in genomic ERα expression within two normal breast cell lines or within three breast tumor cell lines. These results showed that the difference in ERα expression between cell lines, normal or cancer, are not caused by genomic DNA amplification but rather transcription regulation. Hence, Slug may be regulating ERα expression through transcriptional mechanism.

Slug is a member of the Snail family C2H2-type zinc finger transcription factors which bind to E-Box (CANNTG DNA sequence) (37) and represses mRNA transcription (38,39). Therefore, we hypothesized that a key mechanism by which Slug decreases ERα mRNA transcription may be through binding to the ERα promoter region. Six E-Boxes were identified around the promoter region (Fig. 4h). Chromatin immunoprecipitation (ChIP) assay was performed to confirm the mechanism of Slug binding function in MDA-MB-231 cells and MCF-TAMR cells. The data showed that Slug directly binds to E-boxes 1, 2 and 5. Slug did not bind to E-box 3, 4 and 6 (Fig. 4g) (similar results were observed for MCF-TAMR) (data not shown). Notably, E-boxes 1, 2 and 5 have similar DNA sequence, CAGNTG, which may be a specific sequence for Slug binding. Results suggest that overexpression of Slug may repress transcription of ERα gene by binding to E-boxes in the ERα promoter region.

### Slug contributes to EMT in breast cancer cell line

Epithelial-to-mesenchymal transition (EMT) is widely documented as playing a key role in cancer progression by converting both normal and cancer epithelial cells into derivatives with more mesenchymal phenotype (40,41). Based on the results that MCF-TAMR has invasive characteristics (Fig. 1g and h) and that Slug is overexpressed in aggressive breast and prostate cancers, we postulated that Slug may also play an important role for EMT in our cancer cell model. To understand the role of Slug in EMT, MCF7 cells were transiently transfected with control plasmid (MCF7/Con) or Slug plasmid (MCF7/Slug) to determine whether ectopic expression can promote increased mesenchymal phenotype in ERα-positive cells. Slug overexpression was sufficient to lead to a marked decrease in ERα expression at both mRNA (data not shown) and protein levels. The epithelial marker E-cadherin protein level was decreased, while mesenchymal markers, Twist and Vimentin, were upregulated (Fig. 5a). Transfection of Slug to MCF7 cells resulted in >5-fold increase in invasion (Fig. 5b and c). Thus, Slug expression in ERα positive MCF7 cells decreases ERα and E-cadherin while concurrently increases mesenchymal characteristics.

Triple-negative (ERα, PR and Her2 negative) breast cancer is frequently highly invasive and metastatic (42). To examine the role of Slug in this invasive phenotype, MDA-MB-231 cells with knockdown of Slug or control ShRNA (MDA/ShCon) were performed (Fig. 5e). Several independent stable ShSlug clones (MDA/ShC1, MDA/ShC2 and MDA/ShC3) expressing varied Slug levels were isolated (Fig. 7i). After Slug knockdown MDA-MB-231 cells changed morphology from mesenchymal-like to epithelial-like (Fig. 5d). Epithelial marker E-cadherin expression was increased while mesenchymal markers Twist and Vimentin expression was decreased (Fig. 5e). ERα mRNA and protein levels were also increased (Figs. 6c and 7h and i). In the invasion assay, knockdown of Slug decreased cell migration >5-fold (Fig. 5f and g). Importantly, Slug knocked down MDA-MB-231 cells also demonstrated decreased cell migration (Fig. 5h). Thus, Slug expression is required for maintenance of mesenchymal phenotype in ERα-negative MDA-MB-231 cells and may play an important role for epithelial-to-mesenchymal transition.

### Slug increases stemness in breast cancer cells

Recently, it has been shown that there is a link in the relationship between EMT and stem-like properties in normal breast and neoplastic cells. Stemness has been shown to be important for tumor initiation and tumorigenesis (2,41). We performed a Matrigel assay to determine if Slug plays a significant role in tumorgenesis. In the MCF7 cell line, Slug overexpression led to an increase in colony number and size, while Slug knockdown in MDA-MB-231 cells displayed decrease in colonial formation size and number (Fig. 6a and b). Transcription factor PCR array was performed comparing MDA/ShCon with MDA/ShSlug2 cell lines to clarify if the knockdown of Slug involved other master transcription factor changes which include stem cell markers. The Slug knockdown resulted in the downregulation of several transcription factors including stem cell markers c-Myc, Sox2 and Oct4 (Fig. 6c). The expression of the key proteins of cancer stem-like characteristics, CD44 and CD24, were also observed. CD44 has been reported as a cell surface marker for some breast and prostate cancer stem-like cells (19,41,43). Furthermore, CD44^+^CD24^−^/low have been correlated with increased metastatic tumor growth in multiple types of cancer (44). The results showed that after knock-down of Slug, CD44 expression was decreased and CD24 was increased (Fig. 6d). The downregulation of CD44 may affect the tumorgenesis and metastasis in MDA-MB-231 cells. In addition, the interaction between Slug with stem cell markers c-Myc, Oct4 and Sox2 were investigated. Slug demonstrated physical interaction with c-Myc and Oct4 (Fig. 6e) but not Sox2 (data not shown). The interaction between these master transcription factors may play an important role in tumorigenesis and merits further investigation.

To further evaluate the impact of the oncogenic properties of Slug, an *in vivo* experiment was performed. MDA-MB-231/ShCon or MDA-MB-231/ShSlug2 cells were utilized to produce separate subcutaneous mammary xenografts in female nude mice. The tumors derived from MDA-MB-231/ShSlug2 were much smaller (74.3% inhibition) than the tumors from MDA-MB-231/ShCon (Fig. 6f and g). The *in vivo* data strongly support the previous *in vitro* data, suggesting that reduced expression of Slug significantly inhibits the mesenchymal nature of MDA-MB-231 cells thereby altering the invasiveness and tumorigenicity.

### Slug contributes to drug resistance in breast cancer cells

Stemness has also been correlated with cancer drug resistance (15,16,45). Tamoxifen is the most common initial treatment prescribed to ERα-positive breast cancer patients and docetaxel is a widely used chemotherapy drug (46). We tested the drug affectivity in our cell lines. As expected, MCF-TAMR showed resistance to docetaxel (Fig. 7a). Overexpression of Slug in MCF7 cells decreased the sensitivity to tamoxifen and docetaxel (Fig. 7b and c). Knockdown of Slug increased the sensitivity to tamoxifen treatment in MCF-TAMR (Fig. 7d). Knockdown of Slug in MDA-MB-231 cells showed increased response to both tamoxifen and docetaxel treatments (Fig. 7e and f). Recent evidence has correlated enhanced EGFR levels with progression to a metastatic phenotype and drug resistance in multiple cancers (40,47), leading us to suggest that Slug may alter the cell survival signaling pathway between ERα with EGFR. Overexpressed Slug in MCF7 cells results in upregulated EGFR and downregulation of ERα (Figs. 7g and 4a). Downregulation of Slug showed decreased EGFR expression in MCF-TAMR and MDA-MB-231 cells (Fig. 7h and i). These findings demonstrate that the Slug possibly contributes to drug resistance by upregulation of EGFR signaling pathway. Fig. 7j demonstrated the potential mechanism for the alteration of cell characteristics by Slug mediated ERα and EGFR expression.

## Discussion

The alteration in ERα expression is an important step in the development and progression of hormone-related cancers, and it influences cancer response to systemic therapy (3,48). Common to breast cancer, ERα also plays a role in development and progression in prostate cancer (28). Losing ERα expression in breast cancer indicates high risk of cancer. ERα is transcriptionally regulated in both normal tissue and in cancer development. However, more studies are necessary to elucidate differences. Slug is a type of Zinc-finger transcription factor that is critical for embryonic development (49). Evidence shows that Slug is overexpressed in multiple types of cancers (17,27). However, little is known as to how Slug contributes to cancer development.

In the present study, we show the ability of Slug to bind E-boxes of ERα promoter region, and thereby to suppress *de novo* ERα synthesis. This represents a new mechanism in which ERα receptor signaling maintains an epithelial phenotype. Thus, the transcription regulatory mechanism of Slug binding to E-boxes in the ERα promoter region controls ERα activation and function. There was a significant correlation between Slug with cancer progression and metastasis in both breast and prostate cancer tissue samples. The biological action of Slug signaling pathway in cancer indicates that Slug could be a clinical target for future cancer therapy. Since a significant amount of mortality results from cancer metastasis; inhibiting Slug could be an excellent therapeutic target for inhibiting metastasis. Our data identified novel actions for Slug in relation to ERα, EMT, tumorigenesis and drug resistance. In addition, increase in EGFR with Slug overexpression resulting in drug resistance and increase in stem-like markers, explains important adaptive pathway for Slug-induced cancer progression and metastasis. Based on these observations we are proposing the pathway scheme shown in Fig. 7j. The paradigm presented here may also apply to other epithelial cells.

In conclusion, earlier studies have shown that Slug is a key transcription factor important during embryonic development, melanoma progression, and cisplatin resistance in ovarian cancer (18,50,51). It has also been shown that co-expression of Slug with Sox9 increases the mammary stem cell capacity in normal breast cells and promotes tumor formation in breast cancer cells (6). In the present study, we uncovered the interaction between Slug and master transcription factors, c-Myc and Oct4. The function of the protein interaction between these three transcription factors should be of interest for future investigations in both normal and cancer biology. These findings also present evidence that Slug overexpression may cause the increase in cancer stem-like cells, EMT, and drug resistance and could possibly be the Achilles’ heel of aggressive lethal cancers.

## Figures and Tables

**Figure 1:** ERα is downregulated in tamoxifen resistant MCF7 (MCF-TAMR) cell line. (a) Tamoxifen resistant (MCF-TAMR) cell line has been established by culture of MCF7 cells in 10% CDS containing 1 μM tamoxifen for 9 months. (b) The effects of tamoxifen on cell viability. MCF7-WT and MCF-TAMR were treated with 0, 1, 3, 10, 30 and 100 μM tamoxifen, and viable cells were counted by a luciferase-based viability assay after 5 days. (c) E2 induction on cell growth. MCF7 and MCF-TAMR were treated with or without E2 or E2^+^ tamoxifen for 24 h. Then cell growth was measured by an MTT assay (d) analysis of nuclear ERα expression in MCF7 and MCF-TAMR cell line. Immunoflourescence staining using ERα antibody (green) and scale bar 15 μm. (e) The ERα-positive cells were counted in both MCF7 and MCF-TAMR lines. (f) Immunoblot of ERα to confirm ERα expression in MCF7 and MCF-TAMR lines. Cell extracts (50 μg) were loaded in each lane, and the membranes were probed with anti-ERα and β-actin antibodies, respectively, to detect the protein. (g) Cell invasion was assessed using the Transwell invasion assay. (h) The number of invaded cells was counted by imaging (error bars indicate SD, n=3 independent experiments).

**Figure 2:** Slug correlated with breast cancer progression. (a) Transcription factor mRNA levels were compared by qRT-PCR in MCF7, MCF7 treated 5 days with 10^−5^ M tamoxifen and MCF-TAMR cell lines. GAPDH was used as a loading control. (b and c) Slug protein expression was analyzed by immunoblot in MCF7, MCF-TAMR and MDA-MB-231 lines. Cell extracts (50 μg) were loaded in each lane, and the membranes were probed with anti-ERα, Slug and β-actin antibodies to detect the respective proteins. (d) Representative examples of Slug protein expression (intensity) in breast cancer tissues from different patients and embedded on microarray (TMA) platform. Each sample was identified by H&E and tissue histologic/pathology classification. The top 2 samples (normal and ductal carcinoma *in situ*) show Slug negative expression in luminal cell nucleus and the bottom 2 samples (invasive ductal carcinoma and metastasis) show Slug positive expression in cell nucleus. Scale bars, 50 μm. (e) IHC assessment of breast cancer cell nuclear Slug expression from TMA was based on the histologic cellular classification (28 patients 35 cores). (f) Representative examples of Slug and ERα protein expression in breast cancer tissue microarray (TMA). Case 1 shows an example of Slug-positive ERα-negative finding. Case 2 shows an example of Slug-negative ERα-positive finding. Scale bars, 50 μm. (g) IHC assessment of breast cancer ERα and Slug protein expression from breast cancer TMA (21 cancer patients 24 cancer cores).

**Figure 3:** Slug correlates with prostate cancer progression. (a) Representative examples of intense Slug protein expression in prostate cancer tissue microarray (TMA) based on the tissue histologic Gleason score classification and metastasis status. From left to right samples show downregulation of ERα and upregulation of Slug. Staining is recorded on a 2-point scale: (−), negative; (+), positive. The white line indicates the tumor area. White arrow indicates the positive stain. White stars indicate non-specific stain. Scale bar, 50 μm. (b) IF assessment of prostate cancer Slug protein expression from prostate cancer TMA based on prostate cancer histologic Gleason score classification and metastasis status (40 patients). (c) IF staining of 3 cases of cancer-specific death. Scale bar, 50 μm.

**Figure 4:** Slug downregulates ERα expression by binding to E-box on ERα promoter region. (a–e) ERα and Slug expression in normal breast cell lines MCF12A and MCF10A, MCF7, transient MCF12A/Slug, transient MCF10A/ShSlug, transient MCF7/Slug and transient MDA-MB-231/ShSlug cell lines. Total protein was extracted using Thermo protein RIPA buffer, and 50 μg protein for each sample was used for immunoblot analysis. (f) Genomic ERα expression comparison by RT-PCR in MCF10A, MCF12A, MCF7, MCF-TAMR and MDA-MB-231 lines. (g) Chromatin immunoprecipitation assays identified Slug binding sites within the proximal promoter region of ERα gene. PCR reaction products from input control DNA, IgG antibody control and Slug antibody pull-down. (h) Sequence of ERα promoter region contains six E-Boxes as indicated.

**Figure 5:** Slug promotes tumor mesenchymal phenotype. (a) Analysis of EMT-associated protein expression by immunoblot. Total protein was extracted using Thermo RIPA buffer from cells treated for 72 h of transient transfection with either Neovector control or Slug plasmid. Proteins (50 μg) from total cell extract for each sample were used for immunoblot. (b and c) Transwell invasion assay of MCF7 cells after 72-h transient transfection with Neovector or Slug plasmid transfection was performed. (b) The image of cell invasion. (c) The percentage of invaded cells by image (error bars indicate SEM; n=3 independent experiments). (d) Morphology image of MDA-MB-231 stably transfected with ShControl vector or ShSlug plasmid. Scale bar, 20 μm. (e) Analysis of EMT-associated protein expression by immunoblot. MDA-MB-231 was stably transfected with ShControl vector or ShSlug plasmid. Total protein from transfected cells was extracted using Thermo RIPA buffer. Protein (50 μg) was loaded for immunoblot analysis. (f and g) Transwell invasion assay of MDA-MB-231/ShCon and MDA-MB-231/ShSlug was performed. (f) The image of cell invasion. (g) The percentage of invaded cells by image (error bars indicate SEM; n=3 independent experiments). (h) Scratch assay shows the reduced motility of MDA-MB-231 cells stably transfected with ShSlug. Scale bars, 100 μm.

**Figure 6:** Slug promotes tumor formation and metastasis. (a) MCF7 cells, after 72-h transient transfection with Neovector control or Slug plasmid, were subjected to Matrigel colony formation assay. The images show the colonies after 2 weeks in culture. (b) MDA-MB-231 cells, stably transfected with ShControl or ShSlug plasmid, were subjected to Matrigel colony formation assay. The images show the colonies after 2 weeks in culture. The MDA-MB-231/ShSlug2 is a single colony selection number 2. Scale bars in a and b represent 200 μm. (c) The mRNA levels of the transcription factors were compared between MDA-MB-231/ShCon and MDA-MB-231/ShSlug2 by qRT-PCR. GAPDH was used as a loading control. (d) The protein expression level of breast CD24 and CD44 in MDA-MB-231/ShCon and MBA-MB-231/ShSlug. Cell extracts (50 μg) were loaded in each lane, and the membranes were probed with anti-CD24, CD44 and β-actin antibodies to detect the protein. (e) Co-immunoprecipitation (co-IP) between Slug with c-Myc and Oct4. Co-IP was performed with anti-Slug and IgG control antibodies followed by immunoblotting with anti c-Myc and Oct4 antibodies. The nuclear extracts were used in the immunoprecipitation step. (f) Tumor growth curves for xenografs arise from implanting 1×10^6^ cells of MDA-MB-231/ShCon and MDA-MB-231/ShSlug2. (g) Images of xenografts that arise from implanting 1×10^6^ cells.

**Figure 7:** Slug contributes to a drug resistance mediated cell survival pathway between ERα and EGFR. (a) The comparison of sensitivity to docetaxel between MCF7 and MCF-TAMR cells. (b and c) The sensitivity to tamoxifen and docetaxel inhibition of MCF7/Neo and MF7/Slug cells. (d) The comparison of sensitivity to tamoxifen between MCF7-TAMR/ShCon and MCF-TAMR/ShSlug. (e and f) The sensitivity to tamoxifen and docetaxel between MDA-MB-231/ShCon and various MDA-MB-231/ShSlug clones. The docetaxel treatments were performed for 48 h. The cell number was counted after 48-h recovery time. The tamoxifen treatments were performed for 5 days. The cell number was counted after 48-h recovery time (error bars indicate SD, n=3 independent experiments). (g) The expression level of EGFR and β-actin in MCF7/Con and MCF7/Slug. Cell protein extracts (50 μg) were loaded in each lane, and the membranes were probed with anti-EGFR, and β-actin antibodies, respectively, to detect the protein. (h) The expression level of Slug, ERα, EGFR, and β-actin in MCF-TAMR/ShCon and MCF-TAMR/ShSlug. Cell protein extracts (50 μg) were loaded in each lane, and the membranes were probed with anti-Slug, ERα, EGFR and β-actin antibodies to detect the protein. (i) The expression level of Slug, ERα, EGFR, Laminin A/C and β-actin in MDA-MB-231/ShCon and MBA-MB231/ShSlug clone 1, 2 and 3. Cell cytoplasm or nuclear protein extracts (50 μg) were loaded in each lane and the membranes were probed with anti-Slug, ERα, EGFR, Laminin A/C and β-actin antibodies to detect the protein. (j) A model showing possible mechanisms for the alteration of cell characteristics by Slug mediated ERα and EGFR expression.

**Table I:** Primer sequences.

Primer	Primer sequence (5′-3′)	Primer	Primer sequence (5′-3′)
ERα E-box 1	F: 5′-ATTTTGCAGAGGAAGAAACTGAG-3′	Snail	F: 5′-CACTATGCCGCGCTCTTC-3′
	R: 5′-CTATATTTAGCAGCTGGGGGAACT-3′		R: 5′-GGTCGTAGGGCTGCTGGAA-3′
ERα E-box 2	F: 5′-GCTCTTCCTATATGTATACCCTGAA-3′	AR	F:5′-TTAAGAGACAGACTGTGAGCCTAGC-3′
	R: 5′-CTGGGGAGGACTACACTGTAAC-3′		R: 5′-TGAATCTTCCACCTACTTCCCTTAC-3′
ERα E-box 3	F: 5′-GTCCTCCAGCACCTTTGTA-3′	Slug	F: 5′-TGGTTGCTTCAAGGACACAT-3′
	R: 5′-ACGGGAGCAAGTGCAGTC-3′		R: 5′-GTTGCAGTGAGGGCAAGAA-3′
ERα E-box 4	F: 5′-CCTGGGACTGCACTTGCT-3′	Twist	F: 5′-AGTCCGCAGTCTTACGAGGAG-3′
	R: 5′-ACCTGGAAAAAGAGCACAGC-3′		R: 5′-TTGAGGGTCTGAATCTTGCTC-3′
ERα E-box 5	F: 5′-GCTGTGCTCTTTTTCCAGGT-3′	c-Myc	F: 5′-CCTCCACTCGGAAGGACTA-3′
	R: 5′-GAGGGTCATGGTCATGGT-3′		R: 5′-AAGCTCCGTTTTAGCTCGT-3′
ERα E-box 6	F: 5′-CCGGTTTCTGAGCCTTCTG-3′	Jun	F: 5′-GAAGGAGGAGCCTCAGAC-3′
	R: 5′-TCCCTTGGATCTGATGCAGT-3′		R: 5′-CGATTCTCTCCAGCTTCCT-3′
GAPDH	F: 5′-CTTTGTCAAGCTCATTTCCTGGTAT-3′	Sox2	R: 5′-ATGACCAAGCCAGCAGATACTT-3′
	R: 5′-AGCACAGGGTACTTTATTGATGGTA-3′		R: 5′-GCTTAGCCTCGTCGATGAAC-3′
β-catenin	F: 5′-GGACACAGCAGCAATTT-3′	Sox9	F: 5′-CACCAGAACTCCAGCTCCT-3′
	R: 5′-CAGCTGCACAAACAATGGA-3′		R: 5′-AGGTCGAGTGAGCTGTGT-3′
ERα	F: 5′-CTACTGTTTGCTCCTAACTTGCTCT-3′	Oct-4	F: 5′-AGAGGCAACCTGGAGAATTT-3′
	R: 5′-ATATGGTCCTTCTCTTCCAGAGACT-3′		R: 5′-CCGGTTACAGAACCACACTC-3′

ERα, estrogen receptor-α; AR, androgen receptor.
